# Analysis of Brain Activity Changes in Patients with Parkinson's Disease Based on Resting-State Functional Magnetic Resonance Imaging

**DOI:** 10.1155/2022/8561351

**Published:** 2022-01-10

**Authors:** Juan Shen, Chao Xu

**Affiliations:** ^1^School of Medical, Yan'an University, Yan'an, Shaanxi 716000, China; ^2^Department of Radiology, Cardiovascular and Cerebrovascular Branch, Affiliated Hospital of Yan'an University, Yan'an, Shaanxi 716000, China

## Abstract

This paper uses resting-state functional magnetic resonance imaging to observe the changes in local consistency of brain activity in patients with Parkinson's disease (PD). Both healthy volunteers and Parkinson's disease patients were scanned for resting brain functional imaging, and the collected raw data were processed using resting functional magnetic resonance data processing toolkit software. This study adopted the use of Regional Homogeneity (ReHo). The postprocessing method of RS-fMRI is to study the spontaneous brain activity changes of patients with Parkinson's disease and cognitive impairment and to explore the changes in the function of their brain regions in the hope of providing help for the treatment of Parkinson's disease cognitive impairment. The results showed that, compared with the normal control group, the brain regions with increased ReHo values in the PD group were the right central anterior gyrus, the right lingual gyrus, the left middle occipital gyrus, and the bilateral anterior cuneiform lobes. The results show that PD patients have abnormal brain nerve activities in the resting state, and these abnormal brain nerve activities may be related to PD cognitive and behavioral dysfunction.

## 1. Introduction

Parkinson's disease (PD) is a common neurodegenerative disease that occurs mostly in middle-aged and elderly people. Among degenerative diseases of the central nervous system, its incidence is second only to Alzheimer's disease (AD) [1]. Relevant epidemiological statistics show that, among the elderly in China over 65 years old, there are about 1700 PD patients per 100,000 people, and the prevalence is even higher in the elderly over 80 years of age [2]. The main clinical motor symptoms are muscle rigidity, bradykinesia, resting tremor, postural gait abnormalities, and so on. The pathological changes in PD patients are mainly neuronal damage in the substantia nigra compact area and abnormal accumulation of Lewy body (LB) in the brain, resulting in a decrease in dopamine content in the brain and an imbalance of dopamine and acetylcholine, causing related clinical motor symptoms [3]. However, the cause of PD-related pathological changes is currently unclear and may be related to factors such as heredity, age, and environment. In addition to motor symptoms, PD often has nonmotor symptoms (NMS), such as cognitive dysfunction, depression, autonomic dysfunction, and sleep disorders. One of the nonmotor symptoms is mild cognitive impairment (PD-MCI) and Parkinson's disease dementia (PDD). PD-MCI not only affects the patient's social function and the quality of life but also causes a huge burden on the family and society [4, 5]. Therefore, early diagnosis and treatment are particularly important. However, the pathophysiological mechanism of PD-MCI is not clear at present.

At present, the rate of misdiagnosis and missed diagnosis of PD is relatively high, and routine imaging examinations are not specific for the diagnosis of PD. In recent years, functional magnetic resonance imaging has developed rapidly, and it has been applied to the study of many diseases of the nervous system, especially the resting-state functional magnetic resonance imaging (RS-fMRI) [6]. MRI (RS-fMRI) research has become a hot spot. RS-fMRI is an imaging technique that explores changes in the function of the whole brain and its functional connections [7]. The imaging principle is as follows: when the activity of neurons in the local brain area increases, it causes an increase in local oxygen consumption. The content of oxyhemoglobin increases, and the content of relative deoxyhemoglobin decreases correspondingly. Deoxyhemoglobin is a paramagnetic substance, which can cause T2 relaxation time to shorten, so T2 strength of the weighted signal is related to the blood in the local brain area [8]. The ratio of oxyhemoglobin to deoxyhemoglobin is proportional, and the larger the ratio, the higher the signal on the *T*_2_ weighted image. Therefore, when the neuron activity in the local brain area increases, the signal on the *T*_2_ weighted image increases and the level of the *T*_2_ weighted image signal can be used to reflect the activity of the neurons in the local brain area.

Based on the current researches focusing on PD motor dysfunction and the relatively few researches on PD nonmotor symptoms and the advantages of resting-state magnetic resonance, this study adopted low-frequency amplitude and local consistency RS-fMRI postprocessing method to study the spontaneous brain activity changes in patients with Parkinson's disease and cognitive impairment and to explore the changes in brain functions, in the hope that it can provide support for the treatment of cognitive impairment in Parkinson's disease. This study will analyze the correlation between the RS-fMR work data and the scores of the Parkinson's State Rating Scale to explore the relationship between brain function and behavioral external performance. The combination of RS-fMR engineering technology and behavioral research is helpful to understand the relationship between various behavioral characteristics and various characteristics of the human brain functional connection group and guide the understanding of the underlying behavioral abnormalities exhibited by various psychological and mental disorders of neural function mechanisms.

## 2. Related Work

According to whether the task is performed during the scan, the research methods are often divided into task-state fMR work and resting-state fMR work. Classical task-state research mostly uses block design or event-related design to induce subjects to perform brain fMR1 scans with a certain stimulus experience [9]. Task-based fMR research requires subjects to closely cooperate with the implementation of the test task. If the subjects' coordination is poor, similar research results will be more difficult to repeat. The rest state fMR work is different. The subjects neither add external stimuli nor perform any tasks and try not to think about any problems. Tension only needs to be in a quiet, closed, and relatively relaxed state for brain function scans. Since the RS-fMRI does not require subjects to perform the corresponding neuropsychological tasks, the collected spontaneous low-frequency activity information is defined [10]. It is the baseline information of brain function, which can reflect the spontaneous functional activities in the basic state of the central nervous system. Because of its simplicity and ease of implementation, the results of each study are highly comparable, which facilitates the comparison and meta-analysis of results between different research units. Diagnosis and treatment evaluation are more realistic indicators.

Many researchers at home and abroad have used different tasks, different data analysis methods, and different groups of people to confirm the existence of a common brain activity network at rest. In 2003, Massimo et al. [11] used fMR functional connectivity analysis and found that the BOLD signal fluctuations in some brain areas in the resting state have a high time correlation. At the same time, they obtained functional connectivity brain activity maps. They attributed the network center to the posterior cingulate cortex. They returned to the posterior cingulate cortex and proved that the network would not be interrupted during simple sensory tasks. Only when complex cognitive tasks appear can this network be interrupted. The default mode network (DMN) is proposed by Jianan et al. [12]; they also concluded that there is orderly brain activity in the human brain at rest. Pei et al. [13] performed fMR scans on normal healthy elderly people and passed the time-course correlation method after detecting the low-frequency fluctuation signal of fMRI data; the default network with cingulate back as the seed zone has been proved to be basically consistent with the default network performance of normal people discovered by Qinglin et al. [14]. The brain areas that make up the default network include the posterior cingulate gyrus, the medial prefrontal lobe, the dorsal thalamus area, the cuneiform lobe, the precuneus, the hippocampus, and some other lobes. They are mainly located in the midline area, indicating that the specific central nervous anatomy is consistent. Constantin et al. [15] used fMRI technology to present language tasks through auditory perception, further testing the hypothesis of the default activity of the human brain in the resting state.

## 3. Analysis of Local Consistency of Patients' Resting Functional Magnetic Resonance

The research on the default network suggests that, in the resting state without external stimuli, there are regular and relatively intense activities in some areas of the brain. This is an important basis and source of neurocognitive activities, which is important for keeping awake and internal and external. The attention and monitoring of the environment play a supporting role. It shows that the human brain is not completely static in the resting state but maintains specific functions. The Qinglin study [14] shows that normal people are not accompanied by any sensory stimulation and movement. Under the premise of reciting numbers silently or performing motor imagination, the glucose metabolism of the lower and outer parts of both sides of the cerebellar hemisphere increases. It suggests that brain oxygen consumption increases during simple thinking and thinking. Measuring the basal metabolism of the human brain in a resting state with closed eyes, awake, and no specific cognitive tasks can reach one-fifth of the total energy consumption of the human body. In patients with Parkinson's state, due to continuous thinking, theoretically, more energy will be consumed. It is speculated that certain brain areas are more active than non-Parkinson's patients.

Regional Homogeneity (ReHo) [15] analysis is used to study the consistency of spontaneous neuronal activity between a voxel and its neighboring voxels in a resting state and is mainly used to understand the differences in local brain activity. It has been widely used in the research of many neuropsychiatric diseases. In this study, ReHo analysis was used to explore whether there are brain regions with increased or decreased activity in patients with Parkinson's state at rest. The principle of resting functional magnetic resonance is shown in Figure 1.

At present, there are many postprocessing methods for resting-state data, which can be divided into two parts: functional differentiation and functional integration. Functional differentiation is mainly to study the change characteristics of a single BOLD signal and the spontaneous activity of a single neuron, while functional integration is to analyze the changes in signals from the perspective of functional connections and interactions between different brain regions. There are various postprocessing methods for functional integration, mainly including the seed point analysis method. The area of interest is selected in advance as the seed point, and the interaction between the seed point and other brain areas of the whole brain and the functional connection changes, as well as independent components analysis methods, multivariate autoregressive models, Granger causality analysis, and so on [16]. All use different postprocessing methods to analyze the interaction between various brain regions and brain networks. The low-frequency amplitude and local consistency algorithm used in this study are the main postprocessing methods of the functional differentiation part. The principle is mainly in the frequency range of 0.01–0.08 H, which reflects the spontaneous activity changes of neurons in the resting state; the strength of ALFF amplitude can reflect the strength of neuronal activity [17]. The local consistency analysis method is a new resting-state functional magnetic resonance data postprocessing method first proposed by Tuovinen et al. [18]. Its theoretical basis is mainly that there is a high degree of voxels in the same brain area when it is activated. The consistency of the time series will change due to changes in task status. Using this similarity in the time series between voxels, the Kendall harmony coefficient can be calculated, and the Kendall harmony coefficient is used to reflect the neuronal activity. The higher the ReHo value, the higher the synergy of neurons in the local brain area. On the contrary, the lower the ReHo value is, the lower the synergy of local neuronal activity is, indicating that the neurons have abnormal activity performance and this synergy is reduced. It may be related to the pathology of the neurons themselves or it may be caused by abnormal interactions between neurons.

The low-frequency amplitude and local consistency algorithm in resting-state functional magnetic resonance imaging have been widely used in neuropsychiatric diseases. Qinglin et al. [14] in the RS-fMRI study on depressive patients pointed out that, compared with the control group, the ReHo values of the left lobe and bilateral occipital lobe of depressed patients were significantly reduced. It suggests that there are spontaneous neuronal activity disorders in the above-mentioned brain areas of depressed patients. At the same time, it is also widely used in Parkinson's disease-related research. For example, Constantin et al. [15] reported on the use of RS-fMRI to study PD patients that the right forehead of PD patients. There are significant reductions in ReHo values in brain areas such as the dorsolateral cortex and the right inferior parietal lobule. In recent years, more and more scholars have paid attention to the research of RS-fMRI on the functional connection and brain network of the human brain; especially, the brain default network (DMN) research is the most extensive. The default network refers to a brain area that is spontaneously activated by people in a nontargeted directional activity and resting state and has a high degree of functional connectivity. Smitha et al. [16] first proposed the default network concept. Later, through research, we also found brain regions similar to human DMN in monkeys, cats, rats, mice, and other animals. DMN is mainly used for rest, “daydreaming,” and mind. Wandering, nonstimulus-independent thinking, and so on are more active. Initial research by Rashmin et al. [17] pointed out that DMN mainly covers the brain areas of the medial prefrontal cortex and the cingulate gyrus, both sides of the parietal and inferior lobules. The study on resting-state fMRI of DMN pointed out that the precuneus lobes including the hippocampus and parahippocampal gyrus also belong to DMN. A variety of neuropsychiatric diseases such as Alzheimer's disease, schizophrenia, and PD are related to DMN; current researches believe that DMN is mainly related to cognitive functions such as internal and external environmental monitoring, self-introspection, emotion, and memory. A large number of studies have confirmed that changes in DMN's spontaneous activities are closely related to cognitive dysfunction. Therefore, some scholars define DMN as a resting activity closely related to cognition.

RS-fMRI can detect abnormal neuronal activity and abnormal brain network connection changes. The low-frequency amplitude and local consistency algorithm use different methodologies to evaluate brain function and changes in spontaneous neuronal activity from different perspectives. At present, the pathophysiological mechanism of PD patients with cognitive impairment cannot be fully clarified, and imaging diagnosis lacks objective and unified standards [18]. However, the functional abnormalities of PD associated with cognitive impairment and other brain-related diseases often occur before clinical symptoms, and the morphological changes appear. RS-fMRI can detect abnormal changes in brain tissue function and brain function connections in patients with PD complicated with cognitive impairment at an earlier stage, and it has great advantages in exploring the early imaging diagnosis and pathophysiological changes of PD with cognitive impairment.

## 4. Data Processing

Use ReHo analysis to find different brain areas. The brain activity area detected by fMR workers is composed of multiple voxels that are adjacent in space, and multiple voxels form a functional block. ReHo assumes that the selected voxel has temporary similarity with adjacent voxels, and the voxels with local consistency show similar changes in the same time series, using Kendall's coefficient concordance (KCC). As an indicator to measure the consistency and similarity between 1 voxel in a functional blob (27 voxels) and other 26 voxels in time series, the KCC value is assigned to this voxel, and its value is between 0 and 1. Each person's fMR work data gets a KCC image, that is, a ReHo image. Divide the ReHo value of each voxel of the whole brain by the mean value of the ReHo value of all voxels in the whole brain to obtain a standardized ReHo graph, and then perform Gaussian smoothing on the normalized ReHo graph with a Gaussian parameter, after smoothing obtaining standardized ReHo graph enters the next step of statistics [19]. The calculation formula of KCC is as follows:

(1) $$\begin{array}{c} V=\sum_{i}R_{i}^{3}-n{\left(\left(n+1\right)\frac{K}{2}\right)}^{2},\\ T=\frac{\left[k^{2}-\left(n^{2}-n\right)\right]}{12},\\ W=\frac{V}{T}. \end{array}$$

*W* refers to the KCC value of the selected voxel, and its value ranges from 0 to 1; *R*_*i*_ refers to the rank sum of the *i-th* time point, where *V* is the mean value of all *R*_*i*_; *K* refers to the number of time series in a clump (*K* *=* 10), that is, the sum of the number of a single voxel at the core and the number of 10 voxels around it in a cube composed of 10 voxels; *n* refers to the rank, as the total number of points, instant points.

### 4.1. ReHo Analysis Application

MRI data were collected from a Siemens Trio 3.0T magnetic resonance imaging system (Siemens Medical Systems, Erlangen, Germany) with an eight-channel phased front coil. At present, a large number of RS-fMR calculation methods have been proposed. From the perspectives of functional differentiation and functional integration, the functional characteristics of the human brain at the three levels of local brain function, functional subsystems, and complete functional connection groups have been investigated. ReHo analysis is an analysis method that examines the characteristics of functional integration and has obvious methodological advantages. One is that it is a kind of noise reduction processing in both the time dimension and the space dimension, so it will show robustness to temporal noise and spatial noise; the other is that it has no specific requirements for sample distribution and has extremely high applicability. The ReHo analysis method can analyze the consistency of the original signal of the whole brain and infer the function of the corresponding brain area by analyzing the consistency of the spontaneous neural activity of the local brain area. ReHo reflects the synchronization of the time series of neuronal activity in the local brain area, and it is not the intensity of neuronal activity. High ReHo in the brain area indicates that the activity synchronization of the brain area is good; on the contrary, it indicates that the activity coordination of the brain area is poor. ReHo abnormality may be the disorder of the interconnection between neurons, suggesting that local generation and regulation mechanism of neuronal synchronization activity is abnormal. Therefore, ReHo is widely used in the research of Chinese and Western medicine for various diseases [20]. Compared with the healthy control group, in patients with Parkinson's disease with single lateral resting tremor, ReHo in the contralateral anterior cuneiform lobe, inferior frontal gyrus, middle frontal gyrus, parietal lobules, and anterior cingulate gyrus in the ReHo area increased; cerebellum ReHo in the calling area is weakened. The ReHo changes of resting tremor indicate the abnormality of the neuron network, and the increase of ReHo value in some brain areas may be the compensatory effect of the basal ganglia dysfunction, which is consistent with the results of some PET/SPELT studies.

## 5. Experimental Results

### 5.1. Parkinson's State Rating Scale Score

In this study, we compared two groups of patients, the total number of each group is 60, and their ages are between 45 and 70. There were 30 males and 30 females in each group. The average scores and standard error of the two groups of Parkinson's State Rating Scale are shown in Figures 2 and 3.

### 5.2. ReHo Difference Brain Areas between the Parkinson Group and the Healthy Control Group

Figure 4 shows the design of the experiments between the Parkinson group and the healthy group.

The pairwise comparison of the correlation coefficients between the seed points showed that there was no significant difference in the functional connection strength between the ROIs between the overthinking group and the healthy control group. The correlation coefficient reflects not only the strength of functional connection but also the direction of functional connection. Although there is no significant difference in the strength of functional connection between ROIs, it can be seen from the mean correlation coefficient that the functional connection in the PD group is negatively correlated, while the corresponding functional connection of the healthy control group is positively correlated.

The cerebellum is connected to the brain stem through the upper, middle, and lower cerebellar feet and then extensively connected to other nerve structures. We found that the tracer retrogrades from the neurons in the area of the prefrontal area of the cerebral cortex to the basal ganglia neurons and the ventral part of the dentate nucleus, and the area is mainly involved in spatial ability cognition. Therefore, the fiber connection between the cerebellum and the basal ganglia not only coordinates motor functions but also participates in cognitive functions. The cerebral cortex also sends out a large number of fibers to reach the cerebellar cortex through the pons. The cerebellar cortex connected with the limbic lobe is involved in emotional and autonomic functions, and the lateral cerebellar cortex connected with the frontal cortex is involved in cognitive and language functions. These studies show that there are fiber connections between the cerebellum and the basal ganglia and limbic system that participate in cognitive, emotional, and autonomic functions. The results of the study of the different brain regions of ReHo showed that the ReHo value of the cerebellum decreased, and the ReHo of the lobe and the lower gyrus increased. Functional connectivity analysis also showed that the cerebellum and the basal ganglia and the cerebellum and the limbic system were negatively correlated.

The neural network connecting the basal ganglia and the prefrontal cortex is a pathway for regulating emotions, and its functional or structural damage can affect emotions, cognitive processes, and motor functions. In other words, in this study, there is a direct or indirect fiber connection between the leaf dominated by the lenticular nucleus in the basal ganglia and the frontal lobe dominated by the frontal cortex. A study of patients with unilateral injury found that the left and right brain areas play different roles in emotional processing, and those with left injury are more prone to depressive symptoms. Studies have shown that patients with major depression have decreased cerebral blood flow and decreased metabolic rate, and this performance is especially dominated by the left frontal area. Although patients with depression and anxiety were excluded from this study, patients with overthinking have involuntary sighs, lack of initiative, and decreased work efficiency. The scores are higher than those of the healthy control group, and their clinical symptoms are less severe than depression. There may be a decline in left frontal lobe function. The study found that when the left frontal lobe is damaged, the right frontal lobe receives information from the left frontal lobe and completes the function of the left frontal lobe with the help of the biological characteristics of the left and right brain commissures. Based on the above data, it is speculated that the left frontal lobe function of patients with overthinking state is abnormal, the compensatory increase causes the right frontal lobe function to increase, and the compensatory increase produces feedback inhibition on the left lobe, making the two performances negatively related.

Figure 5 shows different brain areas of ReHo between the Parkinson group and the healthy control group.

Through the ReHo analysis, this study found for the first time that, under the premise of Alphasim correction, *P* < 0.05, the ReHo value of the left cerebellum of patients with Parkinson's state decreased; that is, the consistency of local brain spontaneous activity decreased. The ReHo value of the lower back of the lateral dissecting body, the lower back cingulate gyrus of the left side, and the upper frontal gyrus of the right increased, indicating that the local brain spontaneous activity increased uniformly. Further research found that the ReHo value of the left inferior cingulate gyrus was positively correlated with the total score of the Parkinson State Rating Scale (*P* < 0.05) and positively correlated with the factor 1 (mental behavior change) score (*P* < 0.05). The ReHo values of the left cerebellum, the left medial lobe, the lower gyrus of the right dissecting body, and the right upper frontal gyrus have no significant correlation with the total scores of the Parkinson State Rating Scale and 5 factors (*P* > 0.05). Compared with the healthy control group, the ReHo value of the left cerebellum was decreased in the Parkinson group, and the ReHo value of the inner side of the left lobe, the lower gyrus of the right umbilical body, the lower posterior cingulate gyrus of the left, and the upper frontal gyrus of the right increased (*P* < 0.05) Alphasim correction (*P* < 0.05).

The decrease in the ReHo value of the left cerebellum in Parkinson's patients is an interesting finding. The traditional view of cerebellar function is to participate in body balance and muscle tone regulation and coordinate voluntary movement, but the results of this study indicate that the cerebellum may also be related to mental and emotional processing. Many evidences indicate that the cerebellum has nonmotor functions, manifested in sensory, cognitive, and emotional aspects. Studies on children have shown that the cerebellum and brain stem play an important role in the early development of emotions. Cerebellar cognitive affective syndrome is a typical cognitive disorder caused by cerebellar injury. Research suggests that normal people are not accompanied by under the premise of any sensory stimulation and movement; when silently reciting numbers or performing motor imagination, the glucose metabolism of the lower lateral parts of the cerebellar hemisphere increases. Further fMR work research shows that, compared with healthy volunteers, the expected response of the cerebellum of depressed patients to noxious stimuli is lower than that of nonnoxious stimuli. In this study, the small and medium brain areas were located on the outside of the left cerebellum, which is consistent with the results of previous studies. The source of afferent fibers received by the cerebellum is complex, not only in the sensorimotor cortex but also in the dorsolateral and medial prefrontal cortex, the frontal lobe speech area, and the parietal lobe. After receiving signals and integrating them, the lateral side of the cerebellum sends out efferent fibers to relay through the thalamus. The posterior projection to the above-mentioned cortex forms a cortex-lateral cerebellar-thalamus-cortical circuit. These cortical areas are connected with the lateral side of the cerebellum. Therefore, the different brain regions of patients with Parkinson's state have their anatomical basis on the lateral side of the cerebellum. The decrease in ReHo value may be related to the ring path negative feedback regulation; a first-episode depression RS-fMRI study using ReHo analysis also found that the cerebellar ReHo value was reduced.

Figure 6 shows that the local consistency of the left cerebellum of Parkinson's patients is lower than that of healthy subjects. Participants have increased local consistency on the inner side of the left leaf, the lower umbilical body on the right, the lower posterior cingulate gyrus on the left, and the upper frontal gyrus on the right. The cross point is the peak point of the different brain areas.

### 5.3. Correlation between the ReHo Value of Different Brain Regions and the Score of Parkinson's State Rating Scale

The difference between the ReHo value of the brain area and the total factor score is shown in Figure 7. It is divided into 5 factors: factor 1 (psychological and behavioral changes), factor 2 (throat discomfort), factor 3 (head and face discomfort), factor 4 (gastrointestinal discomfort), and factor 5 (neck, shoulder, and limb discomfort). Calculate the total score and each factor score, respectively.

Pearson correlation analysis showed that the ReHo value of the left inferior posterior cingulate gyrus was significantly positively correlated with the total factor score (*P* < 0.05); the ReHo values of the left cerebellum, left inner lobe, right inferior umbilical gyrus, and right superior frontal gyrus were not significantly correlated with total factor scores (*P* > 0.05).

In the PD group, the ReHo values of the right anterior gyrus, right lingual gyrus, left middle occipital gyrus, and bilateral anterior cuneiform lobes were increased; in the right middle frontal gyrus, left inferior temporal gyrus, right middle temporal gyrus, and left olfactory, the ReHo values of the cortex, the right parahippocampal gyrus, the right talus cortex, and the left angular gyrus decreased. Run analysis on the MATLAB platform to import the original data of the anatomical map and the functional map, perform image preprocessing, including time correction, head movement correction, registration, standardization, and smoothing, then determine the activation area (ROL) of the cerebral cortex, convert the data match to the spatial brain map coordinate system to determine the Brodmann (BA) cortical activation zone, and finally superimpose it with the anatomical map, as shown in Figure 8.

As shown in Figure 9, PD is a degenerative disease of the nervous system that easily invades the elderly. It mainly affects the patient's motor function and can cause dementia, becoming one of the main diseases that endanger the health of the elderly. The fMRI technology has become a noninvasive, noninvasive, and precise positioning method for the study of PD brain function. It makes the research of live experimental imaging in neurophysiology and pathophysiology a reality. The fMRI in the resting state means that the subject does not need to complete a specific recognition task and is the spontaneous activity state of the human brain when it is awake. ReHo is a data postprocessing method used to analyze resting-state fMRI data, using the strong similarity (or synchronization) characteristics of the voxel BOLD signal in the active brain area, which can be used without any prior information; detecting the brain area that is continuously active in the resting state is one of the methods for analyzing the slow-wave oscillation characteristics of the local brain area. ReHo detects the brain function by analyzing the similarity of the BOLD signal fluctuations of multiple adjacent voxels in the same time series. The degree of similarity reflects the degree of consistency of neuronal activity in the local brain area, not the intensity of neuronal activity. The decrease of ReHo in a local brain area can indicate a decrease in the consistency of neuronal activity, suggesting that there may be functional abnormalities in this brain area, and it may be that the interconnection between neurons is disturbed.

A large number of pieces of literature [20] on functional brain imaging studies have found that the precuneus is related to many high-level cognitive functions, such as episodic memory, self-related information processing, and various aspects of consciousness. The left middle occipital gyrus may be related to recognition memory, and the talar cortex is related to mental image processing. The central anterior gyrus is mainly responsible for the initiation and execution of movement. This is consistent with the increase in the central anterior gyrus ReHo value in this study in the PD group. The lingual gyrus is considered to be related to dreaming and vision, and it plays an important role in vocabulary recognition. Previous studies have shown that PD patients have changes in visual spatial ability. The angular gyrus is located above the Wernicke area, at the parietal-occipital junction, and is an important joint area in the back of the brain. If the angular gyrus is excised, the visual image of the word will lose contact with the auditory image, and it will cause dyslexia, causing hearing-visual aphasia. The patient loses contact between seeing the object and hearing the sound of the object name and therefore cannot understand the meaning of words. A large number of previous studies [21] have shown that PD patients have the problem of loss of smell. The reduction of ReHo in the limbic system such as the parahippocampal gyrus is believed to be closely related to the cognitive dysfunction of PD. Using voxel-based morphometry (VBM), the cortical atrophy of PD patients mainly appears in the limbic system and prefrontal lobe, and it is considered that it is closely related to the development of PD into PD dementia. This study also shows that the increase of ReHo value means that the consistency of local neuron activity increases, which may be a compensatory response after the appearance of PD cortical damage, while the decrease of ReHo value means that the consistency of local neuron activity decreases, which implies that this brain area may have functional abnormalities or it may be that the interconnection between neurons is disturbed.

## 6. Conclusion

This study found that PD patients have abnormal brain nerve activity at rest. These abnormal brain nerve activities may be related to PD cognitive and behavioral dysfunction. In patients with Parkinson's disease, the local consistency of the left cerebellum is reduced, and the local consistency of the left side lobe, the right lower gyrus, the left lower posterior cingulate gyrus, and the right upper frontal gyrus is higher. Among them, the ReHo value of the left inferior posterior cingulate gyrus was significantly positively correlated with factor 1 of the Parkinson's State Scale (psychological and behavioral changes). It reflects that there are local brain dysfunctions in patients with Parkinson's at rest. These brain areas are mainly related to emotion, cognition, and gastrointestinal function, indicating that Parkinson's patients may have potential recognition in addition to psychoemotional and gastrointestinal dysfunction. The reduced activity of the frontal lobe, parietal lobe, part of the lobes, the cingulate gyrus, right thalamus, right caudate nucleus, and other brain areas in patients with PD cognitive impairment is related to the cognitive impairment of PD patients. The increased activity of some frontal lobes, cerebellum, and other brain regions may be a manifestation of compensatory cognitive function. RS-fMRI can detect abnormal changes in brain function activities at an early stage, which may provide a new image for early recognition of PD patients learn methods. This study did not conduct a stratified study based on the severity of the disease. This study preliminarily shows that patients with mild Parkinson's state do not have functional connectivity changes, but mainly local dysfunction; as the disease worsens, there are gradually obvious functional connectivity changes. Therefore, expanding the sample size can achieve stratified research, which is beneficial to in-depth study of brain function changes with disease progression and its mechanisms.

## Figures and Tables

**Figure 1:** Principle of resting functional magnetic resonance.

**Figure 2:** Average Parkinson's status rating scale scores in the Parkinson group and the healthy control group.

**Figure 3:** Standard error of Parkinson's status rating scale scores in two groups.

**Figure 4:** Resting-state fMRI experiments between two groups.

**Figure 5:** ReHo difference between Parkinson's group and healthy control group.

**Figure 6:** ReHo map of the different brain regions between the Parkinson group and the healthy control group.

**Figure 7:** Correlation between ReHo value of different brain regions and total factor score.

**Figure 8:** The activation area of the cerebral cortex in the spatial brain Atlas coordinate system.

**Figure 9:** ReHo two-sample *t*-test of the PD group and the normal control group.

## Data Availability

The data used to support the findings of this study are available from the corresponding author upon request.
